RETRACTED

# Prevalence and Associated Factors of Peer Victimization (Bullying) among Grades 7 and 8 Middle School Students in Kuwait

**DOI:** 10.1155/2017/2862360

**Published:** 2017-02-28

**Authors:** Ahmad J. Abdulsalam, Abdullah E. Al Daihani, Konstantinos Francis

**Affiliations:** ^1^Kuwaiti Board of Physical Medicine and Rehabilitation, Physical Medicine and Rehabilitation Hospital, Andalous, Kuwait; ^2^Department of Pediatrics, Mubarak Al-Kabeer Hospital, Jabriya, Kuwait; ^3^Almanara Child Psychiatry Unit, Kuwait Centre for Mental Health, Sabah Health Region, Kuwait; ^4^Athens University, Athens, Greece

## Abstract

*Background*. Peer victimization (bullying) is a universal phenomenon with detrimental effects. The aim of this study is to determine the prevalence and factors of bullying among grades 7 and 8 middle school students in Kuwait.* Methods*. The study is a cross-sectional study that includes a sample of 989 7th and 8th grade middle school students randomly selected from schools. The Revised Olweus Bully/Victim Questionnaire was used to measure different forms of bullying. After adjusting for confounding, logistic regression identified the significant associated factors related to bullying.* Results*. Prevalence of bullying was 30.2 with 95% CI 27.4 to 33.2% (3.5% bullies, 18.9% victims, 7.8% bully victims). Children with physical disabilities and one or both non-Kuwaiti parents or children with divorced/widowed parents were more prone to be victims. Most victims and bullies were found to be current smokers. Bullies were mostly in the fail/fair final school grade category, whereas victims performed better. The logistic regression showed that male gender (adjusted odds ration = 1.671, *p* = 0.004), grade 8 student (adjusted odds ratio = 1.650, *p* = 0.004), and student with physical disabilities (adjusted odds ratio = 1.675, *p* = 0.003), were independently associated with bullying behavior.* Conclusions*. There is a need for a school-wide professional intervention program and improvement in the students' adjustment to school environment to control bullying behavior.

## 1. Introduction

Peer victimization or bullying is a repeated aggressive or threatening behavior between peers of unequal size or power, not including teasing in a friendly or playful way [1]. Adolescent bullying takes six forms: verbal, physical, cyber, sexual, racial, and relational bullying [2].

The prevalence of bullying ranges from 6.3% among girls in Sweden to 41.4% among boys in Lithuania [3], with Nansel et al. reporting 30% of students in USA being involved in moderate to frequent bullying: 13.0% bullies, 10.6% victims, and 6.3% bully victims [4]. Fleming and Jacobsen reported that the prevalence of bullying among middle school students in United Arab Emirates was 20% and in Oman 39% [5]. In their meta-analysis of 80 studies providing a total sample of 335,500 youths, Modecki et al. reported mean prevalence rates of 35% for traditional bullying involvement and 15% for cyberbullying [6]. Finally, in a recent published study in Kuwait, the prevalence of bullying in 9th and 10th grade was reported to range, depending on the type of bullying, between 41,6 and 71,1% among boys and between 10 and 81,4% among girls, whilst victimization between 46,2 and 87,9% and between 42,7 and 80,8%, respectively [7]. The discrepancies in the prevalence among the studies could be attributed both to cultural factors and to different definitions and measures employed, and thus caution should be exercised in interpreting them.

RETRACTED

Bullying is associated with social, physical, and mental factors. In general, boys are more likely than girls to be bullies, victims, or both [8, 9]. Although boys and girls may be equally likely to be bullied through calling mean names, teasing, and deliberate exclusion from other students, boys are more likely to receive threats and be physically bullied [10]. The prevalence of bullying and the rate of victimization most probably decline with age [11].

Children are at an increased risk to be involved in bullying if they have difficulties in academic achievement and school adjustment [1, 12] and if they are socially isolated [13], coming from a single parent family [14], having older brothers [15], physically weaker [16], or with a physical disability, such as sight, hearing, walking, or speech problems [13]. On the other hand, positive parental practices are a protective factor for adolescents to be involved in bullying and victimization; having plenty of close friends was found to be negatively related to victimization, whilst adolescents identified as bullies were found to be less socially isolated [12].

Both parties, bullies and bully victims, may have serious, long lasting problems in their life [17]. Bullies and victims are more likely to smoke and have difficulty in making new friends [2, 18]. Kids who bully others are more likely to engage in violent and risky behaviors into adulthood including abusing alcohol and drugs, dropping out of school, having criminal convictions, and engaging in abusive relationships [19]. Children who are being victimized often develop psychological difficulties including social separation and loneliness [20], psychosomatic symptoms and hyperactivity [21], anxiety and social phobia [22], depression and suicidal ideation [23], fear of going to school, and low self-esteem [24]. Bullying can also affect academic achievement [4]. Thus, it is imperative that these consequences are addressed at a younger age, so as their impact on adolescents will be alleviated.

RETRACTED

The aim of this cross-sectional study was to estimate the size of the bullying problem in Kuwait and to investigate the factors associated with it, specifically for the local population. These data can be used to plan an effective and comprehensive antibullying intervention tailored to the specific factors pertaining to the problem in our society. It can also be used to offer data for the study of the phenomenon across cultures, as the bulk of the current literature derives from western societies.

Although a study on bullying behaviors in Kuwait was recently published reporting on prevalence and gender differences in slightly older children than from our sample [7], our study used a different and widely accepted instrument [25] that allows a more meaningful comparison with the international data, as the definitions and measurement can account for large discrepancies in prevalence rates [6]. Furthermore, the previous studies done about bullying in Kuwait did not assess cyberbullying, a relatively new and of increasing importance form of bullying. Finally, apart from gender differences, Alsaleh's study did not address any other factors associated with the behavior.

## 2. Methods

### 2.1. Study Design, Participants, and Procedures

Children in Kuwait attend governmental schools (mostly locals), foreign communities (e.g., Indian and Pakistani) schools (expatriates), and private schools (mixed). Since, for the age group of our study, that is, 12–14 years of age, Kuwaitis form almost 75% of the country population [26] we decided to focus first on this part of the country population, and thus to public schools only. Hence, an approval of the Ministry of Education and their ethical committee regarding the involvement of human participants in the study was sought.

The target population was intermediate school boys and girls at the seventh and eighth grade in public schools in three (out of six) selected governorates of the country: the urban Capital, the rural Al-Ahmadi, and the suburban governorate of Hawalli. With a multistage stratified random cluster sampling method, we randomly selected 5 intermediate schools for males and 5 intermediate schools for females using a table for each governorate, and then from each school, one class was randomly selected from grade 7 and another class from grade 8. All students in the selected classes were included in the study as clusters.

Sample size was estimated based on type 1 error (*α*) of 0.05 and power 0.9 (type two error, *β* = 0.1) and a prevalence of involvement in bullying is 20% similar to that of the culturally close to Kuwait, United Arab Emirates [5], as the Kuwaiti study [7] had not been published at that time. The estimated sample size needed was 961 and to compensate for nonrespondent the sample size was increased to 1000.

RETRACTED

After obtaining permission from the Ministry of Education and the administration of each selected school, informed consent was also obtained from each student. After a standard definition of bullying was given, students were asked to complete a self-administered questionnaire. To ensure confidentiality and the highest possible honesty in their answers the questionnaires were filled in anonymously and without the presence of the classroom teachers. This study was conducted in January 2016.

### 2.2. Instrument

The study questionnaire had 3 sections. Section 1 (question 1 to 10) covered sociodemographic characteristics. Section 2 (question 11 to 17) was adapted from the Revised Olweus Bully/Victim Questionnaire [27] with the author's permission. The Olweus Bully Questionnaire has been widely used to classify adolescents to various categories of bullying behavior during the last year [2]. It also assesses the reactions of others to the situation, for example, “How often do other students try to put a stop to it when a student is being bullied at school?” or “Has any person at home contacted the school to try to stop you from being bullied in the past year?” and where bullying is taking place (“Where have you been bullied?”) with multiple options. Some of the questions pertaining to bullying circumstances were omitted due to time restrictions put by the Ministry of Education and so were the questions for sexual and racial bullying due to cultural restrictions [28]. In addition, cyberbullying is clearly defined beforehand and then investigated in this section with questions that pertained the use of electronic communication to bully a person, typically by sending messages of an intimidating or threatening nature. The 5-point scale (1 = never; 2 = once or twice; 3 = 2 or 3 times a month; 4 = about once a week; 5 = several times a week) was kept and the cut-off of 3 was used to categorize each type of bullying as (a) involved in bullying others only (bullies), (b) involved in being bullied only (victims), (c) involved in both bullying others and being bullied (bully victims), and (d) not involved at all in any of the various forms of bullying [29]. Translation to Arabic from English and independent back translation were performed in order to ensure translation equivalence.

Section 3 (questions 18 to 21) was developed by the first two authors (Ahmad J. Abdulsalam & Abdullah E. Al Daihani) after an extensive review of the current literature on bullying and pertained potential factors associated with bullying, including information about final grade, number of close friends, frequency of smoking, and physical disabilities. Students who reported to smoke at least 1 cigarette per week were categorized as smokers, according to the cut-off point recommended by Bauman and Phongsavan [30]. It also comprised a question (Number 22) assessing student adjustment to school, with seven items, rated on a 5-point scale (1 = strongly disagree; 2 = disagree; 3 = I do not know; 4 = agree; 5 = strongly agree). Those who scored 4 or 5 were categorized as not adjusted to school.

RETRACTED

The questionnaire was pretested on 10 students from 7th and 8th grade in order to assess the clarity of the questions to students and estimate the time needed to answer the whole questionnaire. On average, a student needed about 15 minutes to complete the questionnaire, and few changes were made according the students' feedbacks.

### 2.3. Statistical Analysis

The Statistical Package for Social Sciences (SPSS Inc., Chicago IL, USA, 2010) version 19 was used for data entry and analysis. The *p* value < 0.05 was used as the cut-off level for statistical significance. Pearson's Chi-square test was used to assess the association between two qualitative variables, and this was replaced by Fisher's exact test if the assumption of Pearson's Chi-square test was violated. The multivariant logistic regression for a binary outcome variable was used to identify the independent determinants for bullying, after adjustment for potential confounders. The dependent variable was binary (0 for uninvolved in bullying; 1 for bully, victim, or bully victim). Independent variables included sociodemographic characteristics, smoking status, school achievement, physical disabilities, and adjustment to school.

## 3. Results

In the present cross-sectional study, 1004 seventh and eighth grade middle school children from schools at three governorates were approached and 989 children accepted to participate and returned a completed questionnaire (response rate: 98.5%). Male : female ratio in our sample was 1 : 1.69 which had lower statistical significant than that reported in the last census for this age group (1 : 0.94), due to the smaller class sizes in the male schools.

In our sample, 299 reported that they have been involved in some form of bullying in the past year. Hence, the prevalence (95% confidence interval) of bullying among the studied group was 30.2% (27.4–33.2). Among these, 3.5% (2.5–4.9) were categorized as bullies, 18.9% (16.3–21.5) as victims, and 7.8% (6.2–9.6) as bully victims. Given the significant association between bullying behavior and gender (*p* < 0.001), with boys being more prevalent in all three categories of bullying but statistically significant only in the “Bullies” category (Table 1), and the nonrepresentative nature of our sample regarding sex distribution, the actual prevalence was adjusted slightly higher at 31.6%.

RETRACTED

Table 1 presents the association of self-reported bullying behavior with all the sociodemographic characteristics recorded here. There was a significant inverse association between school grade and bullying behavior (*p* = 0.027) with the prevalence of being victim decreasing between the 7th and the 8th grade. Non-Kuwaiti children were more liable to be victims than Kuwaiti children (36.6% versus 18.1%, *p* = 0.022). Similarly, the proportions of being a bully, a victim, or a bully victim were significantly higher among children whom one of their parents was non-Kuwaiti (*p* < 0.001). Significantly higher proportion of children with divorced/widowed parents reported being involved in a form of bullying than children with regular married parents (*p* = 0.014), especially as bullies (7.1% versus 3.1%).

Governorate of residence was associated with bullying behavior (Pearson's Chi-square, *p* < 0.001). Significantly higher proportion of students living in Hawalli reported to be victims (22.8%) or bully victims (8.2%) versus 13.3% and 6.9%, respectively, for students living in the Capital. Students living in Al-Ahmadi governorate reported the lowest prevalence in various types of bullying. Number of siblings and order among siblings were not significantly associated with bullying behavior (data not reported in Table 1).

Table 2 depicts the association of bullying behavior with school achievement, smoking status, number of class friends, and disability status. There was a significant association between students' final grade last year and bullying behavior (Pearson's Chi-square, *p* = 0.023). The lowest proportion of bullies (1.7%) was in the “excellent” category. Victims performed better than bullies since 17.6% of them were in the “excellent” category. However, 15.4% of the “fail/fair” categories were victims. Besides, there was significant association between smoking status of children and bullying behavior (Fisher's exact test, *p* < 0.001). Among smokers, 28.6% were bullies or victims. However, no significant association was found between bullying and the number of friends. Almost one-third (30.2%) of asthmatic students reported to be victims in the past year, and only 6.7% reported to be bullies (*p* < 0.001). Similarly, 40.7% of students with walking problems reported to be victims (*p* < 0.001), followed by students with obesity (29.7% victims, *p* = 0.011), hearing problems (26.9%, *p* = 0.039), digestive problems (27.8%, *p* = 0.025), eye problems (23.9%, *p* = 0.021), and diabetes mellitus (20.7%, *p* = 0.03).

RETRACTED

Surprisingly, relatively high proportion of teachers (41.3% in case of male students and 56% in case of female students) never or rarely tried to prevent a bullying incident, with only 28% in case of male students and 18.3% in case of females stopping it always or often. Similarly, other students also fail to act protectively in bullying cases with around half of them never or rarely intervening and only 29.5% of the boys and 22.2% of the girls always or often intervening when their classmates are bullied. Moreover, 54.7% of male students and 68.8% of female students reported that no person at home contacted the school to try to stop them being bullied at school. The above figures become more alarming by the fact that bullied victims inform about their situation only in 1/3 of the cases the teacher and school, less than half their parents, and in more than half of the cases their friends. The majority of both males (56.6%) and females (46.7%) reported that they have been bullied at class with the teacher present, followed by physical education class, hallways, and playground.

Table 3 shows the prevalence of bullying behavior (bully, victim, and bully victim) within each form of bullying (verbal, physical, relational, and cyber) according to sociodemographic characteristics. Significantly higher proportion of male students was involved in physical, verbal, and relational bullying than females (*p* < 0.001), with more males being bullies in all subcategories and victims in physical and relational ones. There was no significant difference in the proportion of cyberbullying between males and females. Non-Kuwaiti students were more liable to be victims in all forms of bullying, but with only verbal and rational bullying reaching statistical significance. Similarly, students that one of their parents is non-Kuwaiti were more vulnerable to be victims than if both parents were Kuwaitis in all subcategories except cyberbullying.

Table 4 presents the significant associated factors with bullying behavior using logistic regression analysis in order to adjust confounding between variables. The dependent variable was binary (0 for uninvolved and 1 for bully, victim, or bully/victim). Independent variables included sociodemographic characteristics, smoking status, school achievement, and physical disabilities. The significant variables which were found independently associated with bullying, after adjusting for confounding were gender, school grade, governorate of residence, and physical disabilities. Being male, in 7th grade, resident of the Hawalli governorate, and with physical disabilities were found to be independent determinants for bullying after adjusting for confounding between variables. Male students were at a higher risk to be bullies or victims in reference to females (adjusted odds ratio = 1.671, 95% CI = 1.177 to 2.372, and *p* = 0.004). Grade 7 students were at higher risk to be involved in bullying than grade 8 students (adjusted odds ratio = 1.650, 95% CI = 1.172 to 2.322, and *p* = 0.004). Residents of the Hawalli governorate were at higher risk to be involved in bullying with reference to Capital governorate residents (adjusted odds ratio = 1.750, 95% CI = 1.122 to 2.729, and *p* = 0.014). In addition, students with physical disabilities were at higher risk of involvement in bullying than those students without physical disabilities (adjusted odds ratio = 1.675, 95% CI = 1.195–2.350, and *p* = 0.003).

RETRACTED

## 4. Discussion

Based on this cross-sectional study, the prevalence rates reported in this study are comparable with those reported in some neighboring Gulf countries such as United Arab Emirates and Oman, which have a similar culture and life style [5]. In addition, the prevalence found (almost one-third) was close to the ones reported also in western countries, for example, for 6–10th grade American students [4], and that of Modecki et al. meta-analysis [6], rendering the bullying problem a universal one.

In comparison to the study done by Alsaleh [7], our prevalence rates for each form of bullying (Table 3) were multiple times lower than the previous study reported. However, our data was closer to that of the Kuwaiti Ministry of Education reports that were mentioned in Alsaleh's paper [7]. These differences can be attributed neither to sampling differences as both studies used similar sampling methods and sizes, nor to the grades difference between the two studies. This is because bullying behaviors tend to peak during early adolescence and then decrease, with the turning point being around the 8th grade [31–33], and thus we would have expected in our study, if any difference, higher prevalence rates. Thus, the only explanation can be the differences in definitions and measurements of bullying that can have a substantial effect on the self-report of such behaviors [6, 34]. For instance, our approach was to clearly define to the participants the bullying act using the triad of characteristics that is most accepted in literature, that is, imbalance of power, repetition of the acts, and intention to hurt [1, 27], which would have yielded more conservative estimates than just asking direct questions [6, 35].

RETRACTED

In our study, male students were more prone to be bullies or victims than female students, whilst in western studies boys tend to be overrepresented among bullies or bully victims but girls are more likely to be victims [2]. This difference could be attributed to the fact that Kuwait has segregated schools for males and females. The nationality either of the child or of his/her parents played an important factor of being a victim, a factor not exclusive for this society [36] and an index of insufficient inclusion of expats in Kuwaiti society. Furthermore, the fact that non-Kuwaiti children or children with one of the parents being non-Kuwaiti are considered minority in government schools (only few small categories of expats have access to public schools, e.g., teacher's children) could have resulted in them being more susceptible to victimization. The same pattern was found for children with divorced/widowed parents, a finding that has also been reported in the literature [37]. This may be attributed to the stressful environment in which children from broken families endure. Moreover, children who were resident in Hawalli governorate reported more involvement in bullying behavior than the other two governorates. This may be because Hawalli is one of the more densely populated governorates, with a large number of non-Kuwaiti residents and with lower mean income according to the last census.

Our results reveal an alarming lenient attitude towards the phenomenon in Kuwaiti society, with teachers and parents not readily reacting to it to protect the victims. This is highlighted by the finding that more bullying is done in the classroom even in the presence of teachers than in the playground, a finding contradictory to what was reported in most studies. A possible explanation would be that since more chances for bullying arise in the classroom and the teachers allow it, more bullying incidence will be noted. In contrast, in countries where teachers take a more strict approach towards minimizing victimization, bullies will be more active outside class, where supervision is less.

Whilst bullies are overrepresented in the group of the lower scholastic achievements, victims and bully victims seem to be equally distributed among the groups, although victims performed better. Whilst there is rather an agreement with the literature that bullies have lower academic performance, possibly for them to have a sense control and balance, it is not clear if victims suffer from the same or not. In our sample both bullies and victims were overrepresented in the group of current smokers, which could reflect the vulnerabilities associated with both behaviors (depression, anxiety, poor performance, social difficulties, etc.). Finally, in accordance with Lowenstein [38] but in contrast with Olweus [39], we found that children with physical disabilities were vulnerable to being bullied by other students. Students with walking problems were more probable to be victims, followed by asthmatics, obese children, and children with hearing problems, digestive problems, eye problems, or diabetes.

RETRACTED

### 4.1. Limitations

Although we provided students with clear definition of bullying to minimize subjectivity, the difference in children's interpretation of the meaning of bullying behavior may have affected our results along with the fact that we relied solely on self-reported data. As the study had a cross-sectional design, inferences of directions of findings are not possible. The gender segregated public school system of the country, also, represents a limitation for this study, as its effect on our results is unknown. The exclusion of private schools and hence the Kuwaiti students who attend them decreases the generalizability of our result for this population. Finally, more research is needed for the non-Kuwaiti part of the population, in private schools and in a wider range of ages, so the authorities will be able to design and implement a countrywide program against bullying.

### 4.2. Conclusions and Implication for School Health

This study showed that bullying represents a serious and common problem among Kuwaiti children that warrants specific measures to be taken, taking into consideration the associated factors indicated here. Given the fact that school teachers were found to be lenient to the bullying phenomenon, a first measure should be the formation of a bullying prevention committee at school. This should include all school personnel and should include the sensitization and education. They should enforce the personnel to be alert in recognizing possible signs that a child is being bullied and to administer protection to the possible victims, especially with girls, expats, and children with disabilities [12]. Taking into account the fact that classmates tend also not to react to the phenomenon, peer involvement appears to be an obvious choice, especially since, as we showed in the study, victims tend to turn to their peers for help [12] and bullying involves a group process [40], although research has not concluded their efficacy yet [1]. Changing attitudes towards bullying through specific class programs can also have an effect [41], whilst general programs tackling attitudes towards the “different” (i.e., the expat, the disabled, and the child from a divorced family) were also shown in this study to be needed in Kuwait. In addition, individual level interventions can also be used like talking to students involved in bullying behavior by the social worker or the school psychologist.

RETRACTED

## Figures and Tables

**Table 1:** Association of bullying behavior with sociodemographic characteristics of 7 and 8 grade middle school students in Kuwait.

	Bullying behavior				
	Uninvolved	Bullies	Victims	Bully victims	*p* ^a^
	(*n* = 690)	(*n* = 35)	(*n* = 187)	(*n* = 187)	
	*n* (%)	*n* (%)	*n* (%)	*n* (%)	
*Gender*					
Male	232 (63.6)	23 (6.3)	76 (20.7)	36 (9.8)	<0.001
Female	458 (73.6)	12 (1.9)	111 (17.8)	41 (6.6)	
*Grade*					
7th	310 (65.4)	17 (3.6)	102 (21.5)	45 (9.5)	0.027
8th	380 (73.8)	18 (3.5)	85 (16.5)	32 (6.2)	
*Nationality of the child*					
Kuwaiti	669 (70.6)	33 (3.5)	172 (18.1)	74 (7.8)	0.022^b^
Non-Kuwaiti	21 (51.2)	2 (4.9)	15 (36.6)	3 (7.3)	
*Nationality of parents*					
Both Kuwaiti	657 (71.3)	29 (3.1)	165 (17.9)	71 (7.7)	<0.001^b^
Only one Kuwaiti	30 (47.6)	5 (7.9)	22 (34.9)	6 (9.5)	
*Parental Marital Status*					
Married	620 (71.3)	27 (3.1)	155 (17.8)	69 (7.9)	0.014
Divorced/widowed	76 (59.3)	8 (7.1)	30 (26.5)	8 (7.1)	
*Governorate of residence*					
Capital	175 (75.1)	11 (4.7)	31 (13.3)	16 (6.9)	<0.001
Hawalli	236 (64.8)	15 (4.1)	83 (22.8)	30 (8.2)	
Al-Ahmadi	227 (75.7)	7 (2.3)	50 (16.7)	16 (5.3)	
Others	47 (55.3)	2 (2.4)	22 (25.9)	14 (16.5)	

(i) % represents row percent.

(ii) *p* values were generated using  ^a^Pearson's Chi-square test and  ^b^Fisher's exact test. Frequencies may not add to the total due to missing values.

**Table 2:** Association of bullying behavior with school achievement, smoking status, number of class friends, and physical disabilities.

	Bullying behavior				*p*
	Uninvolved	Bullies	Victims	Bully victims	
	*n* (%)	*n* (%)	*n* (%)	*n* (%)	
*Final grade*					
<70% (Fail/fair)	43 (66.2)	6 (9.2)	10 (15.4)	6 (9.2)	0.018
70–79% (Good)	119 (67.6)	4 (2.3)	32 (18.2)	21 (11.9)	
80–89% (Very good)	260 (67.5)	19 (4.9)	81 (21.0)	25 (6.5)	
90–100 (Excellent)	359 (73.6)	6 (1.7)	62 (17.6)	25 (7.1)	
*Smoking Status*					
Nonsmoker	668 (70.3)	29 (3.1)	179 (18.8)	74 (7.8)	*p* < 0.001
Smoker	8 (38.1)	6 (28.6)	6 (28.6)	1 (4.5)	
*Number of close friends*					
<3	109 (67.7)	74 (7.8)	33 (20.5)	14 (8.7)	0.452
3–5	173 (69.5)	1 (4.5)	48 (19.3)	23 (9.2)	
≥6	371 (71.1)	24 (4.6)	92 (17.6)	35 (6.7)	
*Physical disability*					
Asthma	80 (53.7)	10 (6.7)	45 (30.2)	14 (9.4)	<0.001
Diabetes mellitus	15 (51.7)	2 (6.9)	6 (20.7)	6 (20.7)	0.030^b^
Obesity	39 (52.7)	4 (5.4)	22 (29.7)	9 (12.2)	0.011
Hearing problems	28 (53.8)	2 (3.8)	14 (26.9)	8 (15.4)	0.039^b^
Eye problems	125 (62.2)	5 (2.5)	48 (23.9)	23 (11.4)	0.021
Walking problems	26 (44.1)	1 (1.7)	24 (40.7)	8 (13.6)	<0.001^b^
Digestive problems	18 (50.0)	3 (8.3)	10 (27.8)	5 (13.9)	0.025^b^
Skin problems	53 (58.9)	4 (4.4)	21 (23.3)	12 (13.3)	0.083
Speech problems	18 (54.5)	2 (6.1)	10 (30.3)	3 (9.1)	0.138^b^
Malformations	11 (57.9)	2 (10.5)	5 (26.3)	1 (5.3)	0.208^b^

(i) % represents row percent.

(ii) *p* Values were generated using Chi-square test and ^b^Fischer's exact test.

(iii) Frequencies may not add to the total due to missing values.

RETRACTED

**Table 3:** Prevalence (%) of bullies, victims, and bully victims within each form of bullying (verbal, physical, relational, and cyber) by sociodemographic characteristics.

	Verbal			Physical			Relational			Cyber		
	Bullies	Victims	B/V	Bullies	Victims	B/V	Bullies	Victims	B/V	Bullies	Victims	B/V
*Gender*												
Male	5.5	16.5	3.0	5.2	12.4	1.9	5.5	11.3	1.9	3.0	4.1	0.6
Female	1.3	14.0	0.5	0.7	7.2	0.2	0.7	8.6	1.0	1.5	4.5	0.5
	*p* < 0.001			*p* < 0.001			*p* < 0.001			*p* = 0.437		
*Grade*												
7th	2.8	16.6	2.2	2.6	10.8	1.3	2.4	11.2	1.7	1.1	6.0	0.6
8th	3.0	13.5	0.8	2.2	7.6	0.4	2.6	8.1	1.0	3.0	2.8	0.4
	*p* = 0.158			*p* = 0.128			*p* = 0.288			*p* = 0.011		
*Nationality of the child*												
Kuwaiti	2.9	14.2	1.4	2.4	8.7	0.9	2.5	9.0	1.4	2.2	4.2	0.5
Non-Kuwaiti	2.4	31.7	2.4	2.5	20.0	0.0	2.4	24.4	0.0	0.0	7.5	0.0
	*p* = 0.019			*p* = 0.121			*p* = 0.033			*p* = 0.622		
*Nationality of parents*												
Both Kuwaiti	2.7	13.9	1.3	2.2	8.2	0.8	2.3	8.5	1.3	2.0	4.0	0.4
One non-Kuwaiti	4.9	31.1	3.3	3.4	23.7	1.7	3.3	26.2	1.6	1.6	9.8	1.6
	*p* = 0.001			*p* = 0.001			*p* < 0.001			*p* = 0.066		
*Marital status of parents*												
Married	2.9	14.0	1.5	2.1	8.3	0.9	2.4	8.7	1.4	2.1	3.9	0.4
Divorced/Widowed	2.7	21.4	0.9	4.5	15.2	0.0	3.6	17.0	0.9	1.9	7.1	1.8
	*p* = 0.224			*p* = 0.035			*p* = 0.033			*p* = 0.076		

(i) % represents row percent.

(ii) B/V = bully victims.

(iii) *p* values were generated using Fisher's exact test.

**Table 4:** Significant associated factors with bullying behavior using logistic regression.

Variable	*n*	Adjusted odds ratio	95% CI	*p*
Gender				
Male	341	1.671	(1.177–2.372)	0.004
Female (reference)	529			
Grade				
7th	425	1.650	(1.172–2.322)	0.004
8th (Reference)	445			
Governorate of residence				
Capital (Reference)	204			
Hawalli	333	1.750	(1.122–2.729)	0.014
Physical Disabilities				
No (reference)	419			
Yes	451	1.675	(1.195–2.350)	0.003
Adjustment to school score	986	0.929	(0.929–0.958)	<0.001

(i) Binary logistic regression: dependent variable (0 for uninvolved and 1 for bully, victim, or bully/victim) and independent variables: sociodemographic variables, smoking, final grade, physical disabilities, adjustment to school, and cohesion with family.

(ii) 95% CI = 95% confidence interval for adjusted odds ratio.
